The article "Prognostic and Immunological Significance of FUNDC1 in Hepatocellular Carcinoma: A Study on TCGA Mining" was retracted in 2023. Reasons: signs of a paper mill; compromised peer review; unreliable results or conclusions.

# Prognostic and Immunological Significance of FUNDC1 in Hepatocellular Carcinoma: A Study on TCGA Mining

**DOI:** 10.1155/2022/8371885

**Published:** 2022-08-16

**Authors:** Yuyin Le, Hui Kong, Xu Gao, Jinxiu Zhu

**Affiliations:** ^1^Department of Oncology Medicine, Fuzhou Pulmonary Hospital of Fujian Province, The Teaching Hospital of Fujian Medical University, Fuzhou City, China; ^2^Fujian Institute of Hematology, Fujian Provincial Key Laboratory on Hematology, Fujian Medical University Union Hospital, China; ^3^Department of Radiology Fuzhou Pulmonary Hospital of Fujian Province, The Teaching Hospital of Fujian Medical University, Fuzhou City, China

## Abstract

**Background:**

Hepatocellular carcinoma (HCC) is an inflammation-related malignancy influenced by the immune microenvironment, such as immune tolerance and evasion. HFUN14 domain-with protein 1 (FUNDC1) is a necessary mitochondrial outer membrane protein, functioning as a receptor for hypoxia-caused mitophagy, which is related to human immunity. The relationship between HCC and FUNDC1 in terms of prognosis and immunology was demonstrated in the current investigation. Even so, the function of FUNDC1 in liver cancer is yet unknown.

**Methods:**

The Cancer Genome Atlas (TCGA) and Gene Expression Omnibus (GEO) datasets were utilized for examining if FUNDC1 expression is associated with clinicopathological characteristics and prognosis. Genetic changes (mutation), DNA methylation, and their relationship with patient prognosis were identified by cBioPortal and MethSurv. Utilizing the Tumor Immune Estimation Resource (TIMER), immune checkpoints, infiltration, and immune cell biomarkers were analyzed. Utilizing the STRING database, the network of protein-protein interactions was created. Using Gene Set Enrichment Analysis, the FUNDC1 biological roles were determined (GSEA).

**Results:**

FUNDC1 elevation was significantly linked with gender (*p* < 0.001), tumor stage (*p* = 0.01349), tumor grade (*p* < 0.001), and alpha-fetoprotein (AFP) (*p* < 0.001) levels in HCC. It was illustrated by ROC curve analysis that FUNDC1 had a significant diagnostic and prognostic value. The FUNDC1 genetic change rate was 0.6%. Four out of 6 DNA methylation CpG sites were associated with the HCC prognosis. FUNDC1 is associated strongly with immune cell infiltration in HCC. Moreover, FUNDC1 was positively related to immune checkpoints such as mutant-allele tumor heterogeneity (MATH) (*p* < 0.001), ploidy (*p* < 0.05), homologous recombination defect (HRD) (*p* < 0.001), and loss of heterozygosity (LOH). GSEA revealed significant FUNDC1 enrichment in the cell cycle, hedgehog, and MAPK signaling pathways.

**Conclusion:**

FUNDC1 is a mitophagy regulator that could be a therapeutic, prognostic, and putative diagnostic biomarker for HCC.

## 1. Introduction

Hepatocellular carcinoma (HCC) is a serious public health concern, responsible for 700,000 fatalities each year globally [1, 2]. Although significant inroads have been achieved for HCC treatment over the last decades, the mortality rates and incidence remain high. Besides, the high recurrence and metastatic rates of HCC account for the dismal prognosis of advanced cases [3, 4]. Over the past few years, immunotherapy has shown remarkable success in treating breast cancer, hepatocellular carcinoma, and other cancers [5, 6]. Recently, research into tumor immunity has gained significant momentum. Interestingly, immunotherapy offers an unprecedented chance to efficiently treat malignancies by inducing the immune system against tumor growth and progression [7]. The study of immune-associated genes and the immune microenvironment of HCC improves our understanding of the tumorigenesis mechanism and can guide drug application or treatment measures [8].

FUN14 domain-with 1 (FUNDC1) is a receptor for hypoxia-induced mitophagy anchored to the outer mitochondrial membrane. Mitochondria are a fundamental component of innate immunity, and mitochondrial dysfunction causes immunological activation and chronic inflammatory diseases, including liver cancer [9]. Nonetheless, little is understood regarding the relationship between mitophagy and inflammation in tumorigenesis, warranting further investigation.

This investigation mapped out the FUNDC1 prognostic landscape in liver cancer by applying databases including the Kaplan–Meier Plotter, Cancer Genome Atlas (TCGA), and GEPIA. Next, the associations between FUNDC1 expression and immune cell biomarkers, immune infiltration degrees, and immune checkpoints were explored utilizing both GEPIA and TIMER databases. Besides, the clinical value of FUNDC1 in liver cancer was estimated by analyzing gene mutation, DNA methylation, and pathways linked with the HCC occurrence and progression.

## 2. Materials and Methods

### 2.1. Comparing the FUNDC1 Expression Degree

On the basis of TCGA and GTEx database, FUNDC1 expression in normal and tumor tissues of 34 types of human cancer was investigated. In LIHC, 374 HCC specimens with normal and HCC tissues (50 for each) with their matched neighboring normal tissues were compared. Besides, the GEO datasets GSE62232 and GSE101685 provided us with the gene expression profiles to explore FUNDC1 expression. FUNDC1 protein expression patterns were identified with the Human Protein Atlas database.

### 2.2. Association Analysis of FUNDC1 and Clinicopathological Features and Prognosis

Association analysis of FUNDC1 with age, tumor stage, grade, and AFP was conducted by applying the R package “ggplot2.” On the basis of FUNDC1 mRNA expression, LIHC patients were grouped into two expression groups (higher and lower), using the optimal expression of FUNDC1 as the cutoff value based on R (version 4.0.5). Using the “chisq-test” package, we further conducted a correlation analysis between FUNDC1 and age, gender, tumor stage, grade, and AFP. Using R package “survival,” Kaplan–Meier plots were generated and conducted to assess patients' prognoses (OS, RFS, and DFS). The clinical data applied were obtained from TCGA.

### 2.3. Analysis of Genetic Change of FUNDC1 in HCC

The hepatocellular carcinomas (INSERM, Nat Genet 2015) and liver hepatocellular carcinoma (TCGA, Firehose Legacy) datasets were analyzed by cBioPortal (https://www.cbioportal.org/). Kaplan–Meier plots were generated, and the importance of the diversity between the survival curves (OS and DFS) was identified by performing a log-rank test, and diversities with *p* < 0.05 were of statistical significance.

### 2.4. FUNDC1 DNA Methylation Information

The MethSurv database explored the DNA methylation locations of FUNDC1 within TCGA database (https://biit.cs.ut.ee/methsurv/). In addition, the prognostic values (OS and DFS) of CpG methylation were evaluated.

### 2.5. Association Analysis of FUNDC1 with Immune Checkpoints and Immune Cell Infiltration

To examine if the FUNDC1 expression is related to the biomarkers and immune cell infiltration in HCC, TIMER was utilized (https://cistrome.shinyapps.io/timer/). Besides, R with the ggplot2 package was employed to evaluate the FUNDC1 expression relationship with immune checkpoints in HCC on the basis of TCGA.

### 2.6. Gene Set Enrichment Analysis

FUNDC1's PPI network information was obtained from the STRING database. The interaction was statistically significant when the protein interaction value exceeded 0.9. Utilizing GSEA, we assessed GO terms and the KEGG pathways using screening criteria (*p* value < 0.05 and a false discovery rate (FDR) < 0.05) to study the potential biological activities of FUNDC1.

### 2.7. Statistical Methods

Statistical analysis was conducted with R (v.4.0.5). The Wilcoxon test or *t*-test was adopted for comparing the differences between groups. Pearson or Spearman correlation tests were adopted to determine the correlations. Survival curves were illustrated using Kaplan–Meier plots and compared with log-rank tests. The differentiation between the survival curves was identified, and a *p* value < 0.05 was statistically significant.

## 3. Results

### 3.1. Pan-Cancer Expression of FUNDC1

By integrating TCGA and GTEx databases, we generated a pan-cancer analysis of FUNDC1 mRNA expression.  Figure 1 demonstrates that in 34 cancer types, FUNDC1 was significantly upregulated by comparing it with the related normal tissues, such as invasive breast carcinoma (BRCA), bladder urothelial carcinoma (BLCA), cholangiocarcinoma (CHOL), head and neck squamous cell carcinoma (HNSC), esophageal carcinoma (ESCA), colon adenocarcinoma (COAD), kidney chromophobe (KICH), liver hepatocellular carcinoma (LIHC), lung squamous cell carcinoma (LUSC), thyroid carcinoma (THCA), lung adenocarcinoma (LUAD), and stomach adenocarcinoma (STAD). Nevertheless, kidney renal clear cell carcinoma (KIRC) and ovarian serous cystadenocarcinoma (OV) showed no significant differences. We also found that FUNDC1 was positively elevated in the normal tissues relative to the kidney renal papillary cell carcinoma (KIRP).

The FUNDC1 upregulation was found in both datasets (GSE101685 and GSE62232) (*p* < 0.01; *p* < 0.05) (Figures 2(a) and 2(b)). In paired and unpaired analyses in TCGA, FUNDC1 was upregulated (Figures 2(c) and 2(d)). In addition, HCC sample immunohistochemical staining revealed that FUNDC1 expression in liver tumor tissue was greater relative to the surrounding normal tissues (Figures 2(e) and 2(f)).

### 3.2. Correlations between FUNDC1 Expression and Prognoses

The expression of FUNDC1 was significantly correlated to the T stage, pathological stage, histologic grade, and AFP (Figures 3(a)–3(d)). Patients with advanced-stage disease expressed a higher level of FUNDC1. Based on the Kaplan–Meier survival test, the greater FUNDC1 expression group displayed a relapse survival (RFS) (*p* = 0.0043), a poor OS (*p* = 0.0036), and a disease-free interval (DFS) (*p* = 0.0075) (Figure 4). FUNDC1 overexpression was linked to poor prognosis.

The diagnostic and prognostic value of FUNDC1 overexpression FUNDC1 expression yielded good diagnostic outcomes in differentiating both normal and tumor tissue (AUC = 0.884), as shown by ROC curve analysis (Figure 5(a)). Survival rates at one, three, and five years were predicted by generating a ROC curve of FUNDC1. The AUC values were more than 0.6, suggesting acceptable diagnostic performance (Figure 5(b)). A nomogram was established by combining clinicopathological parameters (such as gender, pathological stage, histological grade, and AFP) and FUNDC1 expression for estimating the 1, 3, and 5 years of survival (Figure 5(c)).

### 3.3. FUNDC1 Genetic Changes in HCC Patients

The current investigation comprised 622 HCC patients. The FUNDC1 genetic change proportion in HCC was 0.6% (Figure 6(a)), and the change rate differed from 0.41 (1/243) to 0.8% (3/377) (Figure 6(b)). Figure 5(c) provides an overview of FUNDC1 changes in HCC. Overall survival (*p* ¼ 0.576) (Figure 6(d)) and disease-free survival (*p* ¼ 0.793) (Figure 6(e)) did not significantly differ as illustrated by log-rank tests and Kaplan–Meier plots between patients with or without variations in FUNDC1.

### 3.4. Methylation of FUNDC1 in HCC Patients

The FUNDC1 methylation of every individual CpG combination was evaluated by the MethSurv tool. 1/6 methylation CpG site, cg02754763, showed the greatest DNA methylation (Figure 7). Prognosis was related to the methylation level of seven CpG sites, including cg01573544, cg02754763, cg07658614, and cg14084176 (*p* < 0.05) (Table 1). The overall survival of patients with low FUNDC1 methylation of these CpG sites was better than individuals with high FUNDC1 methylation.

### 3.5. Immune Cell Infiltration and FUNDC1 Expression Relationship

For examining the link between FUNDC1 expression, immune cell infiltration (CD8+ T cells, B cells, CD4+ T cells, DCs, neutrophils, and macrophages), and tumor purity, TIMER was adopted. A positive relation was detected between the FUNDC1 expression and the degree of B cell infiltration (*r* = 0.429, *p* = 8.38*e* − 17), macrophages (*r* = 0.513, *p* = 2.89*e* − 24), neutrophils (*r* = 0.457, *p* = 3.63*e* − 19), DCs (*r* = 0.448, *p* = 3.59*e* − 18), CD8+ T cells (*r* = 0.336, *p* = 1.71*e* − 10), and CD4+ T cells (*r* = 0.391, *p* = 4.80*e* − 14) in HCC but no correlation with tumor purity (*r* = −0.027, *p* = 6.15*e* − 01) (Figure 8).

### 3.6. Association between FUNDC1 Expression and Biomarkers of Immune Cells in HCC

The association between FUNDC1 expression and biomarkers of immune cells in HCC was identified by applying the TIMER database for investigating the FUNDC1 impact on the tumor immune microenvironment (Figure 9). There was a statistically significant link between FUNDC1 and the following biomarkers: CD8+ T cell (CD8A and CD8B), B cell (CD19 and CD38), M2 macrophage (CSF1R/CD115), M1 macrophage (IRF5), other T cell subsets (Tfh, Th1, Th2, Th9, Th17, Th22, and Treg), natural killer cell (XCL1), TAM (PDCD1LG2, CD80, and TLR7), dendritic cell (CD1C and ITGAX), and neutrophil (ITGAM and FUT4) in HCC. A positive association between immune cell infiltration and HSPA4 was substantiated by these results.

### 3.7. Association between FUNDC1 Expression and Immune Checkpoints in HCC

The FUNDC1 association with mutant-allele tumor heterogeneity (MATH), ploidy, homologous recombination defect (HRD), and loss of heterozygosity (LOH) was evaluated in TCGA and TIMER databases. Between FUNDC1 and the checkpoints mentioned, there was a statistically significant relation (Figures 10(a) and 10(b)).

### 3.8. GO and KEGG Pathway Analyses

Using the STRING database, we established the FUNDC1 PPI network. The top hub genes (SGSTM1, MAP1LC3B, MAP1LC3A, GABARAPL2, ULK2, HSPA8, ULK1, FUNDC2, and HSPA2) were chosen based on their connection degree (Figure 10(a)). Significantly enriched cellular components, biological processes, and molecular functions (*p* < 0.05) were identified during GO enrichment analysis (Figure 10(b)). Significant enrichment of FUNDC1-associated genes was demonstrated in the autophagy pathway (regulation of inflammatory cell), antigen processing and presentation, and signaling pathways, comprising the MAPK signaling pathway and hedgehog signaling pathway (Figure 10(c)). FUNDC1 expression positively correlated with SQSTM1 (Figure 10(d)) and MAP1LC3B (Figure 10(g)) in HCC patients (*r* = 0.107, *p* < 0.001; *r* = 0.34, *p* < 0.001). There was also a correlation between the SQSTM1 and MAP1LC3B upregulation in HCC and the poor prognosis (*p* < 0.001) (Figures 10(e), 10(f), 10(h), and 10(i)).

Anticipated signaling pathways and functional annotations are shown in Figures 11(a)–11(i).

Current evidence suggests that hepatocellular carcinoma (HCC) represents 80%–90% of primary liver cancers [10]. As the leading reason for cancer-specific mortality, HCC ranks 4th globally among cancer-related causes of death [11–13]. Liver cancer is typically driven by chronic inflammation; immune cells are core players in the liver cancer microenvironment and display complex crosstalk with cancer cells [14]. FUNDC1 is critical for human immunity by mitophagy [15, 16]. Nevertheless, the FUNDC1 mechanism in liver cancer is still unknown. Establishing the prognostic significance of FUNDC1 in liver cancer and the association between immune infiltration and FUNDC1 expression was the purpose of the current investigation.

This research substantiated overexpression of FUNDC1 in HCC tissues relative to normal tissues utilizing TCGA and GEO databases. There was a significant link between the FUNDC1 expression and the tumor stage, T stage, AFP level, and tumor grade, which indicated that greater FUNDC1 expression was closely associated with advanced-stage disease. Moreover, ROC curve analysis showed that FUNDC1 yields a good predictive value for the prognosis for HCC.

It is widely acknowledged that gene mutations often lead to poor outcomes. However, in HCC, we found that FUNDC1 genetic alterations were only 0.6%. We also found that genetic alteration is not correlated to the prognosis (OS and DFS). DNA methylation is a prevalent epigenetic process in several types of cancer. The association between FUNDC1 DNA methylation degrees and the prognoses of HCC was investigated. Hypermethylation of six CpG places was related to a worse OS, and cg02754763 showed the greatest DNA methylation levels. They investigate the biological roles of HCC high FUNDC1 expression shown in Figure 12.

Patients with HCC, particularly those with advanced disease, have few treatment choices. HCC is well established to be inflammation-associated, and the immune response plays a vital part in carcinogenesis in HCC. [17] Hence, immune checkpoint inhibitors (ICIs) have the potential to suppress immune reactions in the liver to inhibit the autoimmune process of HCC. An increasing body of evidence suggests that several immunotherapy methods, such as DC-based treatments and immune checkpoint inhibitors, are effective against HCCs, suggesting the significance of immunotherapy for HCC [18–21]. To the best of our knowledge, no molecular biomarkers associated with immunotherapy are currently available for patients with advanced HCC [22, 23]. Accordingly, further research on novel biomarkers to anticipate the ICI therapeutic efficiency in HCC is warranted [24, 25]. Herein, we also found a positive correlation between FUNDC1 and immune cell infiltration level such as T cells (CD8+ and CD4+), B cells, neutrophils, dendritic cells, and macrophages and biomarkers of these cells.

KEGG pathway enrichment analysis displayed that FUNDC1 was enriched in biological processes such as mitophagy, autophagy, and immune processes such as antigen processing and presentation. Moreover, FUNDC1 interacts with SQSTM1 and MAP1LC3B genes to promote the development of HCC. Overexpression of SQSTM1 and MAP1LC3B in HCC also correlated with poor prognosis. Consistently, there is a rich literature that suggests that both MAP1LC3B/LC3B and SQSTM1 are autophagy markers [26–28]. Results of the present study demonstrate that FUNDC1, SQSTM1, and MAP1LC3B have a synergistic function in immune regulation.

FUNDC1 and relevant genes were revealed by GO enrichment analysis to be enriched in functions such as biological processing, cellular component, and protein binding. These results corroborated the effect of FUNDC1 on HCC and the association between FUNDC1 and immune regulation in HCC.

## 4. Conclusions

In conclusion, FUNDC1 has huge prospects for clinical use as an indicator for liver cancer. The diagnostic and prognostic values of FUNDC1 should be more comprehensively investigated by in vivo and in vitro studies. FUNDC1 is closely linked to immune infiltration during the oncogenesis of liver cancer.

## Figures and Tables

**Figure 1:** Pan-cancer expression of FUNDC1. FUNDC1 expression in 34 kinds of normal and cancerous tissues (TCGA and GTEx normal data in comparison with TCGA cancer data), 000*p* < 0.001; ns: no statistical difference.

**Figure 2:** FUNDC1 overexpression in HCC. The volcano plot and histogram showed that FUNDC1 expression was lower in the normal tissue in GSE101685 and GSE62232 datasets relative to HCC (*p* < 0.001) (a, b). Depending on TCGA dataset, which consisted of (c) 374 HCC tissues and 50 normal liver tissues and (d) 50 HCC tissues and their matched neighboring normal liver tissues, the FUNDC1 expression was greater in HCC (*p* < 0.001). HCC sample immunohistochemical staining revealed that the FUNDC1 expression in tumor tissues was greater if compared to the surrounding normal liver tissues (e, f).

**Figure 3:** FUNDC1 expression in relation to the HCC stage. The FUNDC1 expression was significantly linked with (a) T stage, (b) pathological stage, (c) histological grade, and (d) AFP level. 0*p* < 0.05 and 000*p* < 0.001.

**Figure 4:** The prognostic impact of FUNDC1 mRNA in HCC patients (Kaplan–Meier plot). The (a) OS, (b) DSS, and (c) PFI survival curves to compare patients with low (blue) and high (red) FUNDC1 expression in HCC were created using *p* < 0.05 as a cutoff.

**Figure 5:** FUNDC1 nomogram model and ROC analysis. (a) The diagnostic ROC curve for differentiating normal from tumor tissue. (b) Time-dependent survival prediction of one-, three-, and five-year survival rates using ROC curve analysis. (c) Models of nomogram incorporating clinicopathological variables and FUNDC1 grades to estimate 1-, 3-, and 5-year survival.

**Figure 6:** Genetic alterations in FUNDC1 in HCC (a). OncoPrint visual overview of modification on a FUNDC1 query (b). TCGA and INSERM overview of changes in FUNDC1 in HCC (c). Kaplan–Meier curves comparing (d) OS and (e) disease-free survival in patients with/without FUNDC1 gene variation.

**Figure 7:** Visualization of the linkage between the methylation level and FUNDC1 expression.

**Figure 8:** Association between immune cell infiltration and FUNDC1 expression in HCC.

**Figure 9:** Analysis of the association between FUNDC1 and immune cell markers in HCC.

**Figure 10:** The link of FUNDC1 expression with (b) CTLA-4 by TCGA database in HCC and (a) PD-1 by TIMER database.

**Figure 11:** Anticipated signaling pathways and functional annotations, FUNDC1-related proteins in HCC are shown by a bubble plot (a). GO term pathway enrichment analyses (b). KEGG pathway enrichment analyses (c). The association between FUNDC1 and SQSTM1 (d). SQSTM1 survival analysis in HCC (e). SQSTM1 recurrence survival analysis in HCC (f). The FUNDC1 and MAP1LC3B correlation (g). MAP1LC3B survival analysis in HCC (h). Recurrence survival analysis of MAP1LC3B in HCC (i).

**Figure 12:** To investigate the biological roles of HCC high FUNDC1 expression. In discussion, GSEA was applied.

**Table 1:** Hypermethylation status influences the HCC prognosis.

CpG	HR	95% CI	*p*
TSS200-Open_Sea-cg01573544	0.541	0.38-0.77	0.00065
TSS1500-Open_Sea-cg02754763	2.457	1.509-4.001	0.000299
TSS200-Open_Sea-cg04565250	1.133	0.801-1.603	0.480738
1stExon-Open_Sea-cg07658614	0.671	0.463-0.971	0.034427
Body-Open_Sea-cg14084176	0.435	0.275-0.689	0.000379
TSS1500-Open_Sea-cg18511445	1.204	0.848-1.707	0.299126

## Data Availability

The data used to support the findings of this study are included within the article.
